The article "Urinary Angiogenin as a Marker for Bladder Cancer: A Meta-Analysis" was retracted in 2024. Reasons: signs of a paper mill; compromised peer review; unreliable results or conclusions.

# Urinary Angiogenin as a Marker for Bladder Cancer: A Meta-Analysis

**DOI:** 10.1155/2021/5557309

**Published:** 2021-04-27

**Authors:** Amir Hossein Aalami, Hossein Abdeahad, Mohammad Mesgari, Thozhukat Sathyapalan, Amirhossein Sahebkar

**Affiliations:** ^1^Department of Biology, Mashhad Branch, Islamic Azad University, Mashhad, Iran; ^2^Department of Nutrition and Integrative Physiology, Collogue of Health, University of Utah, Salt Lake City, UT, USA; ^3^Department of Biology, Faculty of Science, Ferdowsi University of Mashhad, Mashhad 9177948974, Iran; ^4^Academic Diabetes, Endocrinology and Metabolism, Hull York Medical School, University of Hull, UK; ^5^Biotechnology Research Center, Pharmaceutical Technology Institute, Mashhad University of Medical Sciences, Mashhad, Iran; ^6^Applied Biomedical Research Center, Mashhad University of Medical Sciences, Mashhad, Iran; ^7^School of Pharmacy, Mashhad University of Medical Sciences, Mashhad, Iran

## Abstract

**Aims:**

Bladder cancer (BCa) is a common cancer in North America and Europe that carries considerable morbidity and mortality. A reliable biomarker for early detection of the bladder is crucial for improving the prognosis of BCA. In this meta-analysis, we examine the diagnostic role of the angiogenin (ANG) protein in patients' urine with bladder neoplasm.

**Methods:**

We performed a systematic literature search using ScienceDirect, Web of Science, PubMed/MEDLINE, Scopus, Google Scholar, and Embase, up to 10^th^ October 2020 databases. Meta-Disc V.1.4 and Comprehensive Meta-Analysis V.2.2 software calculated the pooled specificity, sensitivity, area under the curve (AUC), diagnostic odds ratio (DOR), positive likelihood ratio (LR^+^), negative likelihood ratio (LR^−^), *Q*^∗^ index, and summary receiver-operating characteristic (SROC) for the role of ANG as a urinary biomarker for BCa patients.

**Results:**

Four case-control studies were included with 656 participants (417 cases and 239 controls) in this meta-analysis. The pooled sensitivity of 0.71 (95% CI: 0.66–0.75), specificity of 0.78 (95% CI: 0.73–0.81), LR^+^ of 3.34 (95% CI: 2.02–5.53), LR^−^ of 0.37 (95% CI: 0.32–0.44), DOR of 9.99 (95% CI: 4.69–21.28), and AUC of 0.789 and *Q*^∗^ index of 0.726 demonstrate acceptable diagnostic precision of ANG in identifying BCa.

**Conclusion:**

This meta-analysis showed that ANG could be a fair biomarker for the diagnosis of BCa patients.

## 1. Introduction

Bladder cancer (BCa) is the 9^th^ most common cancer globally. The prevalence of BCa is increasing around the world, especially in developed countries [1]. About 3% of current cancer diagnoses and about 2.1% of cancer deaths are attributed to urinary bladder cancer [2]. Around 550,000 new BCa was diagnosed globally in 2018 [3]. In men, BCa ranks sixth in terms of prevalence (around 425,000) and ninth in terms of mortality, while it has a lower prevalence among women (more than 125.000) and ranks seventeenth in terms of mortality [4]. The incidence rate per year is 9.6 per 100,000 men and 2.4 per 100,000 women globally [3]. Geographically, the highest incidence of BCa is found in North America, Europe, Israel, Syria, Egypt, and Turkey [4]. BCa is the sixth most common cancer in Iran [5, 6]. The prevalence of BCa appears to be low in Southeast Asia (excluding Japan), India, South Africa, and Mexico [4]. Several risk factors for BCa have been reported [7], including male sex [8], age [9], smoking [10], alcohol drinking, genetic hereditary, red meat, obesity, pathogens, and environmental contamination, including chlorinated hydrocarbons, polycyclic aromatic hydrocarbons [11], aromatic amines [12], nitrate and nitrite [13], and heavy metals such as mercury and arsenic metals [14, 15]. BCa rarely appears before 45 years and most often appears in the later years of life, with an average age of 69 years for men and 71 years for women [9]. BCa in male patients is around four times higher than in women. Besides, over the last decade, BCa in men has increased by 25% more than in women [16].

The article "Urinary Angiogenin as a Marker for Bladder Cancer: A Meta-Analysis" was retracted in 2024. Reasons: signs of a paper mill; compromised peer review; unreliable results or conclusions.

Noninvasive tools for diagnosis or prediction of BCa have been broadly examined in recent years. Today, urine tests and urinary cytology (UC) tests are used as the primary diagnostic markers of bladder cancer. Biochemical and molecular investigations of blood and urine make a liquid biopsy that could suggest new approaches for prevention, monitoring, and diagnosis [17]. Biomarkers are conceptions driven to present a sweeping landscape of a specific human biological system [18]. These biomarkers include different molecules such as fluorescence in situ hybridization (FISH), nuclear matrix protein number 22 (NMP22), bladder tumor antigen (BTA stat, BTA TRAK), immunocyte/uCyt+, and cytokeratins (CK-18, CK-20, and CYFRA 21-1) which can be used as urinary tumor markers [19, 20]. However, there are some drawbacks for these markers. For instance, the UC accuracy is limited and can be impeded by urinary tract infections, nephrolithiasis, and intravesical instillation therapy [21]. Due to the low sensitivity and specificity in diagnostic of BCa, BTA is not recommended as a routine screening method [22]. The patients may present with various symptoms before the diagnosis of bladder cancer (BCa). In the early stages, many patients do not even express any complaints. Bladder neoplasms can present with bleeding since angiogenesis has an influential role in tumor growth [23–27]. In this regard, angiogenin can be considered a fair tumor marker for BCa. One of the first clinical demonstrators of biomarker-driven BCa to higher clinical achievement was angiogenin (ANG), followed by other pathology progress and beyond [28].

The article "Urinary Angiogenin as a Marker for Bladder Cancer: A Meta-Analysis" was retracted in 2024. Reasons: signs of a paper mill; compromised peer review; unreliable results or conclusions.

Angiogenin (ANG or RNAse 5) is a vascular growth factor and a member of the vertebrate-specific secreted RNase A (EC 3.1.27.5) [29]. ANG contains a single-chain protein including 123 amino acids [30], with 14.4 kDa weight [31], defined through two *α*-helices, seven *β*-sheets, and three disulfide bonds. The gene encoding ANG is located on chromosome 14q11.2 [32]. ANG is the first human tumor-derived protein to develop blood vessels' growth, and it supported the Folkman's hypothesis of tumor growth is angiogenesis-dependent [33, 34]. ANG is a potent angiogenic compound compared to most of other angiogenic agents [35]. Indeed, ANG has been suggested as an approved factor for angiogenesis caused by different angiogenic factors, including vascular endothelial growth factor (VEGF), basic fibroblast growth factor (bFGF), epidermal growth factor (EGF), and acidic fibroblast growth factor (aFGF) [36].

ANG is involved in many cellular processes essential to cell growth and survival [37, 38], inflammation [39], hematopoietic regeneration [40–42], reproduction [43], neuroprotection [44], host defense, innate immune reactions [45], bactericidal effects [46], antioxidant activity [47], wound healing [48], and tumorigenesis [49]. Tumorigenesis is a multistage process that involves genetic and epigenetic changes in tumor cells and selectively supports tumor microenvironment. The available data show that ANG affects almost all tumor formation stages, including tumor cell survival, tumor cell proliferation, migration and invasion of tumor cells, and angiogenesis [35].

Previous studies have revealed the association between ANG and BCa. Accordingly, ANG levels could be useful in the early detection of BCa. Regarding the limitation of available publications, we conducted this meta-analysis to evaluate the role of ANG in the BCa and understand the ability of this biomarker for the diagnosis of bladder cancer.

## 2. Materials and Methods

### 2.1. Search Strategy

This meta-analysis was performed according to the preferred reporting items for systematic reviews and meta-analyses “PRISMA for Diagnostic Test Accuracy” guidelines (Supplementary Table 1) [50]. AH. A, H. A, M. M, and A. S conducted a systematic literature search in various databases, including ScienceDirect, Web of Science, PubMed/MEDLINE, Scopus, Google Scholar, and Embase, up to 10^th^ October 2020. The search keywords such as Angiogenin, ANG, Urinary Bladder cancer; carcinoma; neoplasm, diagnostic tumor marker, “area under the curve” (AUC), ROC curve, sensitivity, and specificity have applied to this research. Moreover, reference lists of target articles were individually searched manually to take additional sources.

The article "Urinary Angiogenin as a Marker for Bladder Cancer: A Meta-Analysis" was retracted in 2024. Reasons: signs of a paper mill; compromised peer review; unreliable results or conclusions.

### 2.2. Eligibility Criteria

The included studies should meet the following criteria: (1) Participants were patients with BCa. (2) Healthy individuals were used as controls. [3] The level of ANG protein in the urine was measured. [4] The diagnostic value or prognostic significance of ANG in BCa patients was assessed. [5] The true-positive, true-negative, false-positive, and false-negative values were reported or obtained by calculating ROC curve data.

The studies were excluded when they were (1) studies without available data or incomplete information, [2] duplicate publications, [3] not written in English, [4] case reports, [5] meta-analyses, [6] letters to editors, [7] comments, [8] reviews, [9] unrelated studies that were eliminated through careful review of the title and abstract of each paper, and [10] articles with only the abstract of the article available.

### 2.3. Data Extraction

AH. A, H. A, and M. M independent reviewers screened the full texts and judged their quality. Conflicts were resolved by discussion to ensure compatibility. The following data was captured in a predesigned form: first author, year of publication, type of sample, sample size, country, method of detection, and results.

### 2.4. Methodological Quality Assessment

The Quality Assessment of Diagnostic Accuracy Studies (QUADAS-2) checklist assessed each study's quality in this paper with nine questions (Supplementary Figure 1, Supplementary Table 2). Each question was answered by ‘high,' ‘low,' or ‘unclear.' Low represents the low risk of bias, while a high or unclear answer represents a high risk of bias. Any conflict between the reviewers was resolved by discussion to reach an agreement.

### 2.5. Statistical Analysis

The diagnostic value of the ANG protein evaluated in patients with BCa was assessed with the random effects model by MetaDisc V.1.4 (Metadisc, Madrid, Spain) and fixed effects model by Comprehensive Meta-Analysis V.2.2 (Biostat, NJ, USA) software to summarize the pooled specificity, sensitivity, positive likelihood ratio (LR^+^), negative likelihood ratio (LR^−^), and diagnostic OR (DOR) with 95% confidence interval (CI), based on the extracted data of true-positive, false-positive, true-negative, and false-negative.

Spearman's rank correlation coefficient is a method that can be used to summarize the strength and direction (negative or positive) of an associated with two variables and also was used to evaluate cut-off threshold effects between sensitivity and specificity. The Cochran's *Q* and *I-*squared (*I*^2^) estimated heterogeneity between studies. The area under the “summary receiver-operating characteristic” (SROC) curves described the overall performance detection method.

The article "Urinary Angiogenin as a Marker for Bladder Cancer: A Meta-Analysis" was retracted in 2024. Reasons: signs of a paper mill; compromised peer review; unreliable results or conclusions.

## 3. Results

### 3.1. Literature Search and Characteristics of Included Studies

Figure 1 shows the flow chart of the literature and study selection. Totally, 455 publications from the databases were collected to assess the diagnostic role of ANG protein in BCa. After removing duplicate studies and those on nonurinary BCa, twenty-five articles were identified and screened by the titles and the abstracts. Of these, thirteen articles were eliminated since they did not fulfill the inclusion and exclusion criteria. After assessing the full texts, eight studies were excluded due to the lack of ROC curve and diagnostic data, or not related to the diagnosis, or the language of the article was not English. Finally, four articles were included in this meta-analysis (Figure 1) [24–27]. The four included studies comprised of 417 patients with BCa. The “enzyme-linked immunosorbent assay” (ELISA) was employed to evaluate the ANG protein in all studies. The characteristics of articles such as AUC, specificity, sensitivity, LR^+^, LR^−^, and sample size are listed in Table 1.

### 3.2. Test of Heterogeneity

Results have shown for metaregression and Spearman rank correlation of sensitivity (1 – specificity) to assess the threshold effect in all test accuracy studies included in the meta-analysis (Table 2). The range between 0.5 and 0.6 interpreted the moderate positive status of the correlation coefficient [51]. Accordingly, the 0.60 of Spearman's correlation coefficient with a *p* value of 0.40 (*p* > 0.05) suggested no heterogeneity from the threshold effect. However, it showed a moderate positive correlation.

The *I*^2^ heterogeneity of sensitivity, specificity, LR^+^, LR^−^, and DOR were 20.8%, 92.1%, 82.7%, 0%, and 77.4%, respectively (Table 3). The heterogeneity based on Cochran's-*Q* were calculated 3.79 (*p* = 0.285) for sensitivity, 37.95 (*p* < 0.0001) for specificity, 17.33 (*p* = 0.001) of positive likelihood ratio, 53.67 (*p* = 0.521) of negative likelihood ratio, and 13.26 (*p* = 0.004) of diagnostic odds ratio, respectively (Table 3).

### 3.3. Diagnostic Value of ANG Protein in Bladder Cancer Patients

The pooled sensitivity and specificity estimated 0.710 (95% CI: 0.662-0.753) and 0.780 (95% CI: 0.736-0.819), respectively (Figures 2(a) and 2(b)). The pooled LR^+^ and LR^−^ were calculated 3.344 (95% CI: 2.021-5.533) and 0.376 (95% CI: 0.320-0.441), respectively (Figures 2(c) and 2(d)). The pooled DOR was calculated at 9.992 (95% CI: 4.691-21.282) based on the random effects model (Figure 2(e)). The AUC curve was 0.83 (Table 3). The ROC plane of sensitivity, specificity, LR^+^, and LR^−^ were shown in Figure 3(a). The SROC represented the diagnostic performance of ANG in BCa patients (Figure 3(b)). The pooled DOR based on the fixed effects model was calculated 7.93 (5.62-11.19) by CMA software (Figure 4). The results demonstrated acceptable diagnostic performance of ANG in BCa patients.

The article "Urinary Angiogenin as a Marker for Bladder Cancer: A Meta-Analysis" was retracted in 2024. Reasons: signs of a paper mill; compromised peer review; unreliable results or conclusions.

## 4. Discussion

In recent years, numerous biomarkers have been reported, particularly those that play a role in cancer development and progression to diagnose BCa [52]. A collection of genetic material derived from urothelial cells can be identified in the urine, including DNA, RNA, microRNAs, and proteins [53].

MicroRNAs (miRs) are small 18-25 nucleotide long nonprotein-coding RNAs that regulate gene expression by pairing to the 3′ untranslated region of their target mRNAs in body fluids as free circulating miRs [54–56]. Urinary miRs can be derived from various specimens—voided urine, urine sediment, or supernatant [57]. Mengual et al. [58] examined the panel of six miRNAs, including miR-187, miR-18a, miR-25, miR-142-3p, miR-140-5p, and miR-204, to assess their role in identifying BCa. According to their report, the sensitivity and specificity were calculated of 85.0% and 87.0% with an AUC of 0.82. Zhang et al. [59] evaluated the diagnostic panel of miR-99a and miR-125b in the urine supernatant in BCa patients. They reported that this panel has 87.0% sensitivity and 81.0% specificity with an AUC of 0.88.

ANG is an effective inducer of angiogenesis *in vivo* and is associated with multiple human neoplasms, diabetic retinopathy, and arthritis. ANG performs a fundamental function in ribosome biogenesis and many cellular processes [60]. However, proteomic profiling of urine has been recommended as an indicative test for BCa [61]. Besides, several biochemical and tumor markers have been identified that could be applied to diagnose BCa with appropriate specificity and sensitivity [62–64]. This meta-analysis demonstrated the role of circulating urinary ANG protein levels for diagnosing BCa. This study showed that ANG level had fair diagnostic efficiency with the AUC of 0.78, 0.710 (95% CI: 0.662-0.753) pooled sensitivity, and 0.780 (95% CI: 0.736-0.819) pooled specificity in BCa patients.

The pooled LR^+^ of 3.344 (2.021-5.533) demonstrated that the diagnostic accuracy of BCa was improved by 3.344-fold with the positive ANG results and the pooled LR-0.376 (0.320-0.441).

The article "Urinary Angiogenin as a Marker for Bladder Cancer: A Meta-Analysis" was retracted in 2024. Reasons: signs of a paper mill; compromised peer review; unreliable results or conclusions.

By merging the LR^+^ and LR^−^, a significant diagnostic index called DOR can be calculated. The higher range of DOR value shows a better diagnostic performance from 0 to infinity limit [65]. In this paper, DOR value for BCa patients accounted for 9.992 (95% CI: 4.691–21.282), which means the urinary ANG has a significant diagnostic effect in these patients. The *Q*^∗^ index is set as the point of indifference on the ROC curve, where the sensitivity and specificity are equal [66]. In this meta-analysis, the *Q*^∗^ index was found to be 0.726, and SROC was 0.789 area under the curve (AUC) for ANG in diagnosing BCa patients. These findings highlight the role of ANG in detecting BCa and potentially could have a crucial role in identifying patients with BCa.

In a meta-analysis reported by Yu et al. [49], the role of serum ANG in various conditions such as diabetes, cardiovascular disease (CVD), neurodegenerative diseases, and cancers was discussed. This study clearly showed that there is not any significant relationship between serum ANG levels in patients suffered from diabetes and neurodegenerative diseases. On the other hand, they noted a significant linkage between serum ANG levels in patients with CVD and cancer compared to the control group. In the subgroup of cancers, the serum ANG concentrations were significantly higher in patients who advanced colorectal cancer (CRC) (*p* = 0.004), acute myelogenous leukemia (AML) (*p* = 0.001), multiple myeloma (MM) (*p* < 0.001), myelodysplastic syndromes (MDSs) (*p* = 0.001), and heart failure (*p* < 0.001) than those in healthy individuals. However, patients with hepatocellular cancer (HCC) (*p* = 0 249), breast cancer (*p* = 0.443), non-Hodgkin lymphomas (NHLs) (*p* = 0.257), and melanoma (*p* = 0.550) did not have significantly higher serum ANG levels than healthy controls. They did not consider bladder cancers in their study. Overall, their study's findings show that serum ANG levels in healthy individuals usually remain in a specific range and are associated with various diseases. Serum ANG levels are not currently a clinical diagnostic marker for the disease. However, significant changes in serum ANG levels in cancers and CVDs suggest that this protein might be involved in the pathogenesis and could be a moderate biomarker for these diseases. Various malignant carcinomas, including prostatic cancer, depend on angiogenesis for growth, invasion, and progression. Pina et al. [67] evaluated the serum levels of ANG as a diagnostic marker in the 252 patients who had prostate cancer. They noted that the median serum ANG levels were significantly higher in prostate cancer patients (*p* = 0.008). They concluded that serum angiogenin levels might help differentiate between cancer and noncancer patients among prostate biopsy candidates.

The article "Urinary Angiogenin as a Marker for Bladder Cancer: A Meta-Analysis" was retracted in 2024. Reasons: signs of a paper mill; compromised peer review; unreliable results or conclusions.

This meta-analysis had some limitations. The major limitation was the small number of studies and participants included because most of the studies were designed for evaluating the diagnosis performance of other biomarkers such as microRNAs. On the other hand, data on the prediction of ANG was also often incompletely reported. Additionally, many trials were of small sample size, with only a few patients assessed by ANG. Hence, the results of this meta-analysis should be confirmed in a study with larger sample size. However, we showed the significant Spearman rank correlation between ANG and BCa patients. Although we demonstrated the diagnostic role of ANG in BCa patients, heterogeneity was low but still present in this analysis. Confounding factors such as gender, race, age, BMI, smoking, comorbidities, and pharmacotherapy may be other causes of heterogeneity that could have affected the results.

This is the first meta-analysis to appraise the urinary ANG marker in patients with BCa and may have clinical value for screening bladder cancer to the best of the authors' knowledge.

Eventually, this meta-analysis showed urinary ANG as a fair and noninvasive tumor marker that can detect BCa patients. Nonetheless, more extensive studies with a larger sample size are needed.

## Figures and Tables

**Figure 1:** Flow chart of the study selection.

**Figure 2:** The sensitivity (a), specificity (b), LR^+^ (c), LR^−^ (d), and DOR (e) forest plots for the diagnosing role of ANG in the bladder carcinoma patients based on the random effects model.

**Figure 3:** The ROC plane curve (a) and SROC (b) for diagnosing the role of ANG in the bladder carcinoma patients based on the random effects model.

**Figure 4:** The diagnostic odds ratio based on the fixed effects model meta-analysis performed with CMA software.

**Table 1:** Comparison of different studies on urinary angiogenin (ANG) as a diagnostic biomarker in bladder cancer.

Author/year	Country	Case	Control	AUC	Sensitivity	Specificity	PPV	NPV	Accuracy	Cut-off	Detection method
Eissa/2004	Egypt	63	46	0.775	75.4%	70.3%	84.9%	80.0%	81.2%	322.7 ng/mg	ELISA
Eissa/2009	Egypt	240	110	0.77	75.2%	69.5%	NR	NR	NR	425.0 pg/mg	ELISA
Shabayek/2014	Egypt	50	20	0.803	66.0%	75.0%	76.74%	63.82%	NR	145.0 pg/ml	ELISA
Urquidi/2012	USA	64	63	0.857	67.0%	97.0%	96.0%	74.0%	86.0%	410.9 pg/ml	ELISA

BCa: bladder cancer; AUC: area under the curve; PPV: positive predictive value; NPV: negative predictive value; NR: not reported; ELISA: enzyme-linked immunosorbent assay.

**Table 2:** Results of the Spearman rank correlation of sensitivity against (1 − specificity) to assess the threshold effect in all test accuracy studies included in meta-analysis for diagnosing ANG in patients with bladder cancer.

Analysis of diagnostic threshold				
Spearman correlation coefficient: 0.600, *p* value = 0.40				
Logit (TPR) vs. logit (FPR)				
Where log represents the natural logarithm.				

Moses' model (*D* = *α* + *βS*)				
Weighted metaregression (inverse variance)				
Variables	Coefficient	Std. error	*T*	*p* value
*α*	1.954	0.254	7.680	0.016
*β* (1)	-0.703	0.252	2.791	0.108
Tau − squared estimate = 0.1007				

Moses' model (*D* = *α* + *βS*)				
Weighted metaregression (study size)				
Variables	Coefficient	Std. error	*T*	*p* value
*α*	1.961	0.246	7.961	0.015
*β* (1)	-0.759	0.174	4.358	
Tau − squared estimate = 0.1840				

TPR: true-positive rate; FPR: false-negative rate, Std. error: standard error; *D* = logit TPR − logit FPR; *S* = logit TPR + logit FPR; *α* is the intercept value; *β* represents the dependence of test accuracy on the threshold.

The article "Urinary Angiogenin as a Marker for Bladder Cancer: A Meta-Analysis" was retracted in 2024. Reasons: signs of a paper mill; compromised peer review; unreliable results or conclusions.

**Table 3:** Pooled AUC, *Q*^∗^ index, sensitivity, specificity, LR^+^, LR^−^, and DOR for diagnosing ANG in the urine of patients with bladder cancer based on the random effects model.

No. studies	AUC	*Q* ^∗^	Variables	Pooled (95% CI)	*I* ^2^ (%)	Cochran's-*Q*	*τ* ^2^	*p* value
4	0.789	0.726	Sensitivity	0.710 (0.662-0.753)	20.8%	3.79	NA	0.285
			Specificity	0.780 (0.736-0.819)	92.1%	37.95	NA	<0.0001
			LR^+^	3.344 (2.021-5.533)	82.7%	17.33	0.197	0.001
			LR^−^	0.376 (0.320-0.441)	0%	53.67	0	0.521
			DOR	9.992 (4.691–21.282)	77.4%	13.26	0.443	0.004

AUC: area under the curve; *I*^2^: *I*-squared; *χ*^2^: Chi-squared; *τ*^2^: tau-squared; NA: not assessed; LR^+^: positive likelihood ratio; LR^−^: negative likelihood ratio; DOR: diagnostic odds ratio; CI: confidence interval. *I*^2^ = 100% × (*Q* − df)/*Q*, where *Q* is the Chi-squared statistic and df is the degree of freedom of *Q* statistic.

## Data Availability

There is no original raw data associated with this systematic review.

## Supplementary Materials

Supplementary Materials Supplementary Table 1: PRISMA-DTA checklist item. Supplementary Figure 1: overall quality assessment of included articles using the QUADAS-2 tool. Supplementary Table 2: results of the QUADAS-2 quality assessment of included studies.
